# The Clinical Value of Thyroid Hormone Levels and Correlation with Severity of Liver Cirrhosis

**DOI:** 10.1155/2022/5365172

**Published:** 2022-06-06

**Authors:** Chang Liu, Li Li, Li Zeng

**Affiliations:** Department of Gastroenterology, The First People's Hospital of Chong Qing Liang Jiang New Area, Chongqing 401121, China

## Abstract

**Background:**

The aims of this study were to expound the effect of thyroid hormone on the occurrence of liver cirrhosis and the severity classification of liver cirrhosis with meta-analysis.

**Methods:**

A comprehensive search of PubMed, EMbase, The Cochrane Library, Web of Science, Google Scholar, CNKI, and WanFang Data databases and reference lists of retrieved articles was performed since the inception of each database until September 2021. Two reviewers independently screened literature, extracted data, and assessed the risk of bias by RevMan 5.3 software. In continuous variable analysis, the standardized mean difference (SMD) and 95% confidence interval (95% CI) were calculated through a random-effect model.

**Results:**

Eighteen case-control studies involving 3336 subjects were included for review. The results of the meta-analysis showed free triiodothyronine (FT3) and free thyroxine (FT4) levels in the liver cirrhosis group were lower than the control group (SMD = −1.29, 95% CI [−1.85, −0.74], *P* < 0.001), (SMD = −0.61, 95% CI [−0.96, −0.26], *P* < 0.001), thyroid-stimulating hormone (TSH) levels in liver cirrhosis group were higher than the control group (SMD = 0.34, 95%CI [0.06, 0.63], *P* < 0.001) and that FT3 levels in Child-Pugh A VS B and Child-Pugh B VS C group were higher than the control group (SMD = 1.08, 95%CI [0.80, 1.37], *P* = 0.008), (SMD = 0.68, 95%CI [0.38, 0.98], *P* < 0.001).

**Conclusions:**

Cirrhosis has decreased FT3 and FT4 levels and increased TSH levels. FT3 levels correlate negatively with the Child-Pugh score, and it is a measure of the severity of liver cirrhosis dysfunction. FT3 serum levels of thyroid hormones are a prognostic marker in liver cirrhosis.

## 1. Background

In the last twenty years, the intricate relations between the thyroid gland and the liver in health and disease have aroused extensive attention. As an important chemical plant of the body, there is a certain correlation between thyroid and liver diseases in clinical diagnosis and laboratory. Thyroiditis, hyperthyroidism, or hypothyroidism can occur in patients with chronic liver disease or liver insufficiency. Patients with abnormal thyroid function, such as hyperthyroidism, may have abnormal liver function examination [1]. The thyroid gland is the largest pure endocrine organ in the body, and the thyroid gland produces hormones needing to be degraded, excreted, and transformed by the liver. Liver disease may affect thyroid function and lead to thyroid metabolic disorder [2]. The type and severity of liver disease play crucial roles in thyroid hormone, which, in turn, is also of great significance to early diagnosis, severity assessment, and treatment of liver disease. Therefore, the correlation between thyroid hormone and liver disease is well studied [3].

The Child-Pugh score system was aimed at predicting mortality in patients with cirrhosis. Then, the patients were divided into three groups: A- good hepatic function, B- moderately impaired hepatic function, and C- advanced hepatic dysfunction. The Child-Pugh score could help to predict the risk of death and liver-related complications in patients with liver disease [4]. It was worthwhile to study cirrhosis Child-Pugh, grade A, B, and C three groups, and serum thyroid hormone indexes. The Child-Pugh score of cirrhosis could evaluate the severity of liver cirrhosis. The results indicated that the higher the Child-Pugh score was, the worse the prognosis of patients with liver cirrhosis would be.

Free triiodothyronine (FT3), free thyroxine (FT4), and thyroid-stimulating hormone (TSH) were the most representative ones of thyroid hormone [5]. Serum FT4 levels remain either normal or slightly low in patients with liver cirrhosis, and serum TSH levels remain normal or slightly raised. The main changes in the determination of plasma thyroid hormone level were the concentration of total T3 and free T3. Up to now, fewer studies have clearly mentioned FT3, FT4, and TSH levels with the severity of liver cirrhosis. There was no meta-analysis to clarify the correlation between the thyroid hormone and the severity of liver cirrhosis. Currently, there is also no meta-analysis about changes in the thyroid hormone with liver cirrhosis. The abnormal thyroid hormone level could be used to judge the severity of patients with liver disease [6]. The aims of this study by integrating data for meta-analysis were: First–Thyroid hormone levels (FT3, FT4, and TSH) in patients with liver cirrhosis. Second–To investigate the relationship between thyroid hormone level and the severity of liver cirrhosis.

## 2. Methods

Our researchers searched PubMed, Embase, The Cochrane Library, Web of Science, Google Scholar, CNKI, and WanFang Data from the inception of each database until September 2021. The search keywords were as follows: (“liver cirrhosis” or “cirrhosis” or “hepatic cirrhosis”), (“thyroid hormone” or “thyroid” or “FT3” or “FT4” or “TSH” or “free triiodothyronine” or “thyroid-stimulating hormone” or “free thyroxine”), and similarly searched for references in the existing literature. Additional citations were sought by analyzing the reference list of all previously selected articles.

### 2.1. Eligibility Criteria

Eligible criteria are as follows: (1) Initial studies discussed the association between thyroid hormone level and liver cirrhosis; (2) Case-control study or nested case-control expressed published journals in English or Chinese. (3) The presentation of the number of positive/negative thyroid hormones (FT3, FT4, and TSH) and liver cirrhosis. (4) The comparison between the control group (healthy persons) and the thyroid hormone level of each Child-Pugh score in patients with cirrhosis.

Exclusion criteria were as follows: (1): Duplicate research reports. (2) Reviews and meta-analyses. (3) Irrelevant literature. (4) The unit of measure could not be converted. (5) The articles that did not provide complete data. (6) Liver cirrhosis was accompanied by serious complications or liver cancer. (7) The control group was not healthy people.

### 2.2. Data Extraction

All data were extracted, and quality was assessed independently using the inclusion and exclusion criteria form designed by our group, with differences resolved by discussion. The following information features were extracted in each study: The first author, year of publication, country, article title, and population; Demographic characteristics of study participants (total number of people in each group), thyroid hormone parameters of cases and controls including the Child-Pugh score; the parameters unit of TSH, FT3, and FT4. The units of relevant data should be unified. We had converted and unified the FT3, FT4, and TSH units according to the international standard units(The FT3 unit: pg/ml, FT4 unit: ng/dl, TSH unit: u IU/ml).

### 2.3. Inclusion of Research Bias Risk Assessment

Two researchers independently screened, sorted, and extracted the data with disagreements discussed, and the consensus was finally reached. The risk of bias in the case-control study was assessed using the New Castle Ottawa scale. Through the selection of research objects, comparability between groups, and exposure factors, 8 items were included in the study, with a full score of 9 points, 0–4 points for low-quality studies, and 5–9 points for high-quality studies.

### 2.4. Statistical Analysis

Analyses were performed using the software Review Manager 5.3. As for extracted data, standardized mean difference (SMD) with 95% CI and the point estimate were calculated using the effect index. The heterogeneity of the included results was analyzed by chi-square test (test level: *α* = 0.10). *I*^2^ was used to evaluate the heterogeneity of results: a fixed effect model was used in *I*^2^ < 50% indicates minor heterogeneity, and a random-effect model was used in *I*^2^ > 50% indicating large heterogeneity. We performed the subgroup study according to different ethnic groups, and there was the Child-Pugh score with liver cirrhosis related to thyroid hormone. Sensitivity analysis was performed to assess the impact of bias risk on the significance of the effect. Funnel charts were used to analyze publication bias, and an asymmetric plot suggested possible publication bias. At this stage, studies with a certain risk of bias were excluded from meta-analysis and were assessed for changes in the overall significance.

## 3. Results

### 3.1. Study Selection

We identified 1461 potentially relevant studies through online and manual search, including 474 relevant Chinese articles and 987 relevant English articles. Then, 1239 studies were excluded by reviewing the titles and abstracts. Screening selected 222 articles' full text with reference to the inclusion criteria and 138 articles for lack of effective data or case-control data. In addition, review articles, case analyses, clinical reviews, guidelines, and animal studies were also excluded (66 articles), and 18 studies were included in the present meta-analysis [7–24]. The relevant data of all included literature is listed in Table 1, thyroid hormone, and Child-Pugh classification of liver cirrhosis are in Table 2. Then, Figure 1 presents the flowchart of the study selection process.

### 3.2. Study Characteristics

A final sample of 3336 participants from different countries was analyzed.18 articles (10 Chinese articles,8 English articles) met the eligibility criteria and were included in the qualitative synthesis articles. These articles consist of 1950 cirrhosis patients and 1386 normal controls (58.5% vs. 41.5% in cirrhosis and noncirrhosis). Geographical areas of the reports were subdivided as follows: Turkey, India, Japan, Belgium, Egypt, Italy, and China. Except for five European populations and one African population, other studies were on Asian peoples. (66.7%) articles with available data were the Child-Pugh score of liver cirrhosis.

### 3.3. Meta-Analysis and Subgroup Analysis

#### 3.3.1. Liver Cirrhosis Patients with FT3, FT4, and TSH Levels Compared with Control Group

FT3 levels in the liver cirrhosis group were lower than the control group (SMD = −1.29, 95% CI [−1.85, −0.74], *P* < 0.001) (Figure 2(a)). FT4 levels in the liver cirrhosis group were lower than the control group (SMD = −0.61, 95% CI [−0.96, −0.26], *P* < 0.001) (Figure 2(b)). TSH levels in the liver cirrhosis group were higher than the control group (SMD = 0.34, 95% CI [0.06, 0.63], *P* < 0.001) (Figure 2(c)). Meta-analysis results were obtained by integrating data to find three groups of heterogeneity (*I*^2^ = 98%, 95%, 93%). The random-effects model was used to calculate the standardized mean difference (SMD) and 95% confidence interval (95%CI). The forest plot results are described in Figure 2.

#### 3.3.2. Subgroup Analyses

We performed a subgroup analysis based on the different ethnic groups: Five European populations and one African population with FT3, FT4, and TSH levels compared with the control group, which involved 850 patients in liver cirrhosis group and 543 in the control group. In Asian race groups, FT3 levels in the liver cirrhosis group were lower than the control group (SMD = −1.33, 95% CI [−2.22, −0.54], *P* < 0.001), and in non-Asian race groups (SMD = −1.17, 95% CI [−1.60, −0.74], *P* < 0.001). With regard to FT4, non-Asian race groups might not be significantly associated with liver cirrhosis (SMD = 0.20, 95% CI [−0.36, 0.77], *P* < 0.001). Then, the results were different in Asian race groups (SMD = −1.00, 95% CI [−1.41, −0.59], *P* < 0.001). To TSH, the pooled SMD of 0.18 with a 95% CI of −0.07 to 0.43 (*I*^2^ = 63%) indicated that it might not be significantly associated with liver cirrhosis, but in Asian race groups, TSH levels in liver cirrhosis group were higher than the control group (SMD = 0.42, 95% CI [0.01, 0.86], *P* < 0.001). The forest plot of subgroup analyses results are described in Figures 3(a)–3(c).

#### 3.3.3. The Child-Pugh Score of Liver Cirrhosis Patients with FT3, FT4, and TSH Level

FT3 levels in Child-Pugh A VS B and Child-Pugh B VS C group were higher than control group (SMD = 1.08, 95% CI [0.80, 1.37], *P* = 0.008), (SMD = 0.68, 95% CI [0.38, 0.98], *P* < 0.001). FT4 and TSH levels were not significantly different between the Child-Pugh score of liver cirrhosis and control group (SMD = 0.22, 95%CI [−0.32, 0.76], *P* < 0.001), (SMD = 0.24, 95% CI [−0.12, 0.59], *P* < 0.001), (SMD = −0.02, 95% CI [−0.18, 0.13], *P* = 0.43), (SMD = −0.11, 95% CI [−0.51, 0.30], *P* < 0.001). The results of all subgroup analyses are shown in Figure 4.

### 3.4. Sensitivity Analyses

Sensitivity analysis was performed to identify potentially influential studies. The results of all individual analysis and subgroup analysis were similar before and after deletion of each included study, suggesting high stability of the meta-analysis results. The significance of the estimated combined SMD was not unduly affected, suggesting that the results were robust.

### 3.5. Bias Diagnostics

The results showed that the distribution of TSH, FT3, and FT4 in the study of liver cirrhosis was symmetrical, which indicated that there was no possibility of publication bias. Similarly, in the Child-Pugh score group, we could see that the funnel plot is symmetrical, indicating that there is no publication bias. The funnel charts are shown in Figure 5.

## 4. Discussion

From chronic hepatitis to cirrhosis, the metabolism of hormones in the liver changed. Abnormal liver function was associated with thyroid function. It was worthy of further study that the change in thyroid hormone level was valuable for predicting the degree of liver injury. The changes in serum thyroid hormone levels in patients with liver cirrhosis were mainly related to the following reasons: (1) After the occurrence of liver cirrhosis; the thyroid would atrophy or even cause degenerative changes in the hormone feedback mechanism, which might affect the secretion and synthesis of thyroid hormone. (2) Liver cirrhosis was usually accompanied by changes in a random internal environment such as blood flow and pH value. Under the feedback mechanism of the body, the T4 transformation function was further blocked, which could lead to the decline of T3 level. (3) Liver cirrhosis puts the body in a state of stress, hypothalamus-pituitary thyroid axis dysfunction, and thyroid hormone regulation decline, which causes the change of serum thyroid hormone levels. (4) The body's energy metabolism was blocked, hypersplenism induced anemia, and Na^+^-K^+^ - ATP activity decreased, which affected the process of iodine uptake and thyroid hormone levels [25–27].

As early as 1974, Chopra [28] showed that in patients with liver cirrhosis serum, T3 levels were decreasing in most cases, but there was no hypothyroidism in clinic Symptoms. Serum FT3 and FT4 were not affected by plasma protein concentration. It could reflect the change of thyroxine in liver cirrhosis. Therefore, the changes of FT3 and FT4 were selected to observe the changes in thyroid hormone in patients with liver cirrhosis in meta-analysis. It was reported in the literature that the levels of FT3 and FT4 were low in patients with liver cirrhosis [29–31]. Then, the study report showed that TSH levels were higher with liver cirrhosis [32, 33]. Our results were consistent with these studies, and the results were reliable. Serum FT3 and FT4 in patients decreased gradually with the aggravation of liver cirrhosis, which was negatively correlated with Child-Pugh grade [34, 35]. But so far, according to the document retrieval results, there has been no meta-analysis report on the relationship between liver cirrhosis and thyroid hormone. Meanwhile, the literature about Child-Pugh score and thyroid hormone in patients with liver cirrhosis was less. In particular, most of the existing literature was Chinese. We integrated the relevant literature and a total of 18 case-control studies involving 3336 subjects concerning this aspect.

Our meta-analysis found that (1) decreased FT3 and FT4 levels were significantly associated with a higher risk of liver cirrhosis; (2) increasing TSH levels were positively associated with the risk of liver cirrhosis, suggesting primary hypothyroidism. (3) The level of FT3 was related to the severity of liver cirrhosis and correlated negatively with the Child-Pugh score. (4) Levels of FT4 and TSH could not decrease with the Child-Pugh grade increased, and the hormone levels of FT4 and TSH could not predict the severity of the liver disease. (5) FT3 level was a reliable index to predict the prognosis of patients with liver cirrhosis. Subgroup analysis based on the different ethnic groups showed that there were differences in some results between the East and the West and between Asian race groups and non-Asian race groups (FT4 and TSH). This might be associated with the fact that our research included more studies on China and Asia.

List the shortcomings of our meta-analysis: First, the meta-analysis covered less than 5000 patients, and small sample studies were more prone to generate heterogeneity. We attempted to explore to give a more conservative estimate of the effect by sensitivity and meta-regression analyses and a random-effects model. Second, the basis of our study on only the published Chinese and English literature might lead to selection bias. Third, there were more studies from Asia than from other regions, and the results could be more suitable for the Asian population. Fourth, there was no uniform standard for hormone level of FT3, FT4, and TSH. Therefore, there would be some deviation in the results due to different methods. In the recent 5 years, there has been almost no attention and concern to designing case-control studies. Fifth, most of the 18 articles included were not classified by the etiology of liver cirrhosis and were lacking in subgroup analysis.

In conclusion, by our meta-analysis and integrating data, this further confirmed the changes of thyroid hormone levels in patients with liver cirrhosis. The detection of serum thyroid hormone could be used to judge the severity of liver cirrhosis and evaluate the prognosis. FT3 levels were correlated negatively with Child-Pugh score, which is a measure of severity of liver cirrhosis dysfunction.

## Figures and Tables

**Figure 1:** Flow diagram of the study screening and selection process.

**Figure 2:** Forest plots of studies investigating FT3 (a), FT4 (b), and TSH (c) with Liver cirrhosis.

**Figure 3:** Forest plots of subgroup analysis based on the ethnic groups. (a) FT3. (b) FT4. (c) TSH.

**Figure 4:** Forest plots of the Child-Pugh score and FT3 hormone levels with liver cirrhosis.

**Figure 5:** The funnel charts of FT3, FT4, and TSH in the study of liver cirrhosis.

**Table 1:** Characteristics of the studies included in the meta-analysis.

Study	Area	Ethnology	Sample size		FT3 (pg/ml)	FT4 (ng/dl)	TSH (uIU/ml)	NOS core (sub)
Shimada 1988	Japan	Asian	Control	40	3.17 ± 0.77	1.86 ± 0.30	2.90 ± 1.40	8
			Cirrhosis	17	2.42 ± 0.76	1.51 ± 0.29	3.20 ± 2.60	

Vincken 2016	Belgium	European	Control	50	3.30 ± 0.45	1.30 ± 0.16	1.77 ± 1.23	8
			Cirrhosis	29	2.80 ± 0.59	1.18 ± 0.19	1.60 ± 0.74	

Sahin 2019	Turkey	European	Control	367	2.95 ± 0.95	0.89 ± 0.74	2.28 ± 5.14	8
			Cirrhosis	577	2.14 ± 0.75	0.86 ± 0.55	2.010 ± 1.59	

Punekar 2021	India	Asian	Control	100	3.13 ± 0.59	1.86 ± 0.36	3.15 ± 1.20	8
			Cirrhosis	100	1.95 ± 0.57	1.27 ± 0.54	4.09 ± 1.70	

Kabbany 2012	Egypt	African	Control	30	3.90 ± 1.00	1.49 ± 0.50	3.50 ± 1.40	7
			Cirrhosis	40	1.90 ± 0.20	1.60 ± 0.40	4.05 ± 1.40	

Bianchi 1991	Italy	European	Control	48	3.25 ± 1.00	0.92 ± 0.22	1.85 ± 0.94	7
			Cirrhosis	118	2.57 ± 1.08	0.87 ± 0.33	2.41 ± 2.96	

Spadaro 2003	Italy	European	Control	13	3.31 ± 0.69	1.24 ± 0.23	1.54 ± 0.73	6
			Cirrhosis	45	2.77 ± 0.79	1.16 ± 0.31	2.10 ± 1.33	

Atalay 2014	Turkey	European	Control	35	3.05 ± 0.59	0.77 ± 0.10	1.41 ± 0.82	6
			Cirrhosis	41	2.32 ± 0.67	1.27 ± 0.28	2.06 ± 1.37	

Qian XF 2020	Chinese	Asian	Control	48	2.96 ± 0.18	0.95 ± 0.01	4.25 ± 0.07	8
			Cirrhosis	60	2.74 ± 0.35	0.35 ± 0.08	4.28 ± 0.10	

Guo ZP 2020	Chinese	Asian	Control	180	2.62 ± 0.59	0.92 ± 0.19	1.96 ± 1.41	7
			Cirrhosis	180	3.38 ± 0.34	0.87 ± 0.11	2.10 ± 0.89	

Wu B 2010	Chinese	Asian	Control	40	4.02 ± 1.36	1.42 ± 0.27	0.35 ± 0.98	7
			Cirrhosis	66	0.91 ± 0.39	0.88 ± 0.13	0.83 ± 0.15	

ZhangDY2012	Chinese	Asian	Control	30	5.52 ± 1.34	1.84 ± 0.29	2.58 ± 0.24	6
			Cirrhosis	128	3.34 ± 1.62	1.12 ± 0.25	3.85 ± 0.32	

Li ZH 2018	Chinese	Asian	Control	50	3.34 ± 0.33	1.18 ± 0.13	2.00 ± 0.74	8
			Cirrhosis	189	2.23 ± 0.44	1.09 ± 0.25	1.94 ± 1.54	

Gu W 2016	Chinese	Asian	Control	129	3.26 ± 0.46	1.29 ± 0.18	2.11 ± 0.89	8
			Cirrhosis	104	2.40 ± 0.62	1.14 ± 0.24	2.45 ± 1.56	

Ge QL 2016	Chinese	Asian	Control	53	2.32 ± 0.84	1.39 ± 0.60	2.69 ± 2.07	8
			Cirrhosis	65	1.96 ± 0.57	1.03 ± 0.71	3.96 ± 2.07	

Wu WW 2019	Chinese	Asian	Control	103	3.25 ± 0.34	0.91 ± 0.11	1.31 ± 2.62	8
			Cirrhosis	121	2.33 ± 0.42	0.78 ± 0.98	1.24 ± 2.92	

Wang YR 2016	Chinese	Asian	Control	30	2.24 ± 1.08	1.45 ± 0.68	5.18 ± 4.6	7
			Cirrhosis	30	1.85 ± 0.90	1.37 ± 0.66	4.33 ± 4.8	

Qi GH 2013	Chinese	Asian	Control	40	2.66 ± 0.52	1.19 ± 0.09	2.20 ± 1.00	7
			Cirrhosis	40	1.81 ± 0.58	0.92 ± 0.27	2.10 ± 1.00	

**Table 2:** Thyroid hormone and Child-Pugh classification of liver cirrhosis.

Study	Sample size		FT3 (pg/ml)	FT4 (ng/dl)	TSH (uIU/ml)
Punekar 2021	Child A	1	1.90 ± 0.10	0.76 ± 0.10	4.41 ± 0.10
	Child B	37	2.20 ± 0.55	1.44 ± 0.54	3.68 ± 1.64
	Child C	62	1.80 ± 0.53	1.17 ± 0.51	4.34 ± 1.71

Spadaro 2003	Child A	15	2.79 ± 0.56	1.05 ± 0.28	1.71 ± 1.61
	Child B	15	2.62 ± 0.75	1.06 ± 0.15	2.68 ± 1.26
	Child C	15	2.84 ± 1.01	1.31 ± 0.36	2.03 ± 1.04

Atalay 2014	Child A	10	2.83 ± 0.56	1.09 ± 0.19	1.79 ± 1.08
	Child B	13	2.34 ± 0.40	1.24 ± 0.18	2.41 ± 1.59
	Child C	18	2.03 ± 0.73	1.40 ± 0.32	1.95 ± 1.36

Qian XF 2020	Child A	20	1.14 ± 0.13	0.45 ± 0.02	4.29 ± 0.11
	Child B	20	0.83 ± 0.17	0.32 ± 0.12	4.30 ± 0.11
	Child C	20	0.38 ± 0.13	0.25 ± 0.12	4.32 ± 0.08

Guo ZP 2020	Child A	85	2.96 ± 0.44	0.84 ± 0.12	2.17 ± 1.56
	Child B	61	2.43 ± 0.39	0.98 ± 0.20	2.02 ± 1.34
	Child C	34	2.14 ± 0.40	1.03 ± 0.19	1.33 ± 0.91

Wu B 2010	Child A	11	1.75 ± 1.16	1.10 ± 0.20	1.34 ± 0.76
	Child B	18	1.10 ± 0.90	0.94 ± 0.13	0.94 ± 0.35
	Child C	37	0.77 ± 1.16	0.71 ± 0.16	0.64 ± 0.89

Zhang DY 2012	Child A	25	5.13 ± 1.45	1.57 ± 0.24	3.42 ± 0.26
	Child B	42	2.82 ± 1.57	0.89 ± 0.27	3.45 ± 0.25
	Child C	61	1.91 ± 1.26	0.72 ± 0.18	4.28 ± 0.46

Li ZH 2018	Child A	36	2.71 ± 0.43	1.01 ± 0.17	1.72 ± 1.18
	Child B	72	2.12 ± 0.50	1.01 ± 0.23	1.68 ± 1.23
	Child C	81	1.98 ± 0.44	1.14 ± 0.24	1.66 ± 1.33

Gu W 2016	Child A	24	2.81 ± 0.64	1.10 ± 0.23	1.98 ± 1.10
	Child B	53	2.36 ± 0.64	1.16 ± 0.25	2.54 ± 1.88
	Child C	27	2.09 ± 0.31	1.11 ± 0.20	2.67 ± 1.09

Ge QL 2016	Child A	19	2.31 ± 0.60	1.14 ± 0.41	3.17 ± 0.21
	Child B	24	1.97 ± 0.37	0.97 ± 0.21	3.46 ± 1.93
	Child C	22	1.61 ± 0.44	0.79 ± 0.25	3.60 ± 2.10

Wu WW 2019	Child A	30	2.77 ± 0.32	0.76 ± 0.94	1.49 ± 3.09
	Child B	34	2.36 ± 0.33	0.91 ± 0.15	0.86 ± 2.76
	Child C	57	1.90 ± 2.31	0.80 ± 1.00	1.11 ± 2.95

Qi GH 2013	Child A	8	2.27 ± 0.45	0.96 ± 0.15	2.50 ± 1.00
	Child B	12	1.81 ± 0.38	0.85 ± 0.16	2.30 ± 1.40
	Child C	20	1.16 ± 0.38	0.80 ± 0.07	2.30 ± 1.40

## Data Availability

The raw data supporting the conclusions of this article can be obtained from the corresponding author upon request.
